# Effect of Tetracycline Antibiotics on Anaerobic Digestion of Chicken Manure Based on Data Mining

**DOI:** 10.1155/2022/6335146

**Published:** 2022-06-15

**Authors:** Haiqi Zhai, Hong Qiang

**Affiliations:** College of Resources and Environment, Northwest A&F University, Yangling 712100, Shanxi, China

## Abstract

Although anaerobic bioengineering treatment of chicken manure has the advantages of low energy consumption, less pollution, and recyclable biomass energy, antibiotics are usually added in the process of modern intensive farming. And antibiotics still exist in feces and pose a threat to human health. Therefore, this study aimed to deeply understand the role of TC in the anaerobic digestion of chicken manure and to analyze the effect of tetracycline antibiotics on the anaerobic digestion of chicken manure based on data mining. In this study, chicken manure was used as raw material for anaerobic fermentation, and the effects of tetracycline (TC) on anaerobic and anaerobic fermentation of chicken manure were compared through batch and sequence experiments. Also, this study analyzes the fermentative transformation to elucidate the effect of TC on anaerobic manure conversion in chicken manure, which further studies the effect of TC on the anaerobic fermentation of chicken manure. The experimental results in this study show that when the TC concentration is 50–150 mg/L, the content of tryptophan and tyrosine proteins in the treatment group is also higher than that in the control group. It shows that at low concentrations (10, 25 mg/L), TC mainly promotes the degradation of LEPS by promoting the dissolution of intracellular substances in the sludge. With the increase of TC concentration (50–300 mg/L), TC mainly promotes the breakdown of the sludge cell membrane by promoting the rupture of the sludge cell membrane, thereby promoting the degradation of LEPS.

## 1. Introduction

While large-scale chicken farming has improved production efficiency, it has also resulted in a large amount of chicken manure being produced in some areas. If these chicken manures are not properly handled, it will bring serious harm to the surrounding environment of the chicken farm. Anaerobic digestion technology can not only degrade organic pollutants but also produce clean energy and organic fertilizers. It is a green and environmentally friendly method of chicken manure treatment and utilization. In order to meet the growing demand, the scale of the poultry industry has continued to expand and the breeding density has continued to increase. Correspondingly, the excrement of laying hens and broilers is also produced in a large amount, resulting in the local area nutrient exceeding the land carrying capacity. About 10,000 chicken farm can produce up to 1.3 tons of manure per day.

The results showed that the TC concentration of 300 mg/L had an inhibitory effect on the microbial regulation mechanism. It provides a theoretical basis for the mechanical application of the anaerobic fertilizer digestion process.

The innovations of this study are as follows: (1) Through the experiment of anaerobic digestion of chicken manure with tetracycline antibiotics and the change in methane produced by anaerobic digestion of chicken manure under different TC concentrations, in this study, by increasing the concentration of TC in stages, the characteristics of anaerobic digestion of TC-contaminated chicken manure were studied, which provided a reference for practical engineering applications. (2) In this study, the changes in methane are produced by anaerobic digestion of chicken manure under different TC concentrations and the experiment of anaerobic digestion of chicken manure. (3) Combined with the analysis of the microbial population structure, the microbiological mechanism of the effect of TC on the anaerobic digestion of chicken manure was elucidated, which provided a theoretical basis for the engineering application of the anaerobic digestion process of TC-contaminated livestock and poultry manure.

## 2. Related Works

Anaerobic monodigestion of chicken manure is applicable as the microbial community becomes acclimated to high TAN concentrations. Recep nder Surmeli studies have shown that acetate-consuming methanogens are adversely affected by TAN and total sulfide concentrations higher than 4000 and 100 mg/l, respectively [1]. The results of Hu's study showed that fipronil had a significant effect on biogas production during CM and CS AD [2]. When pig manure is used as a substrate in a biogas plant, it may have an impact on anaerobic digestion. The purpose of Wang's study was to investigate the effects of CTC and Cu on the anaerobic digestion of batches of pig manure in order to better estimate and control the risks of antibiotics and heavy metals on anaerobic digestion. The results showed that a high concentration of CTC had no significant effect on cumulative gas production (*P* > 0.05), but it seriously delayed the daily peak gas production [3]. Chuenchart W study used a small anaerobic continuous stirred tank reactor (CSTR) system under wet conditions with a working volume of 87 L and a total solids content of 10%. The organic loading rate is higher in the anaerobic co-digestion system due to the synergistic effect of microorganisms, buffer capacity, and nutrients [4]. To reduce the occurrence of antibiotic resistance genes in manure, Wu investigated the changes in ARGs and mobile genetic elements (MGEs) during co-composting of chicken manure with Chinese herbal medicine residues for 46 days. Among *β*-lactam resistance genes, the relationship between blaOXA1 and composting days was the strongest (*P* = 0.016), and the removal rate was 78.63%[5]. Y Lu investigated the effect of adding sulfur and Thiobacillus 1904 on N conversion during composting [6]. It is critical to remove antibiotics before livestock manure is exposed to the environment. Anaerobic digestion (AD) is an effective technology for processing livestock manure. Fu et al. showed that the use of tetracycline reduced the methane yield by 8.8%, alleviating its inhibitory effect [7]. Yin F's found that the effect of combined antibiotics on AD varies with individual antibiotics, the negative impact of combined antibiotics on AD is less, and methane production increases with decreasing antibiotic concentration [8].

## 3. Anaerobic Digestion of Chicken Manure with Tetracycline Antibiotics

### 3.1. Anaerobic Digestion and Tetracycline

At the same time, the digestive juice produced by anaerobic digestion can also be used as fertilizer for agricultural production [9, 10]. Tetracycline (TC) is a broad-spectrum antibacterial agent and one of the most frequently used antibiotics in aquaculture and livestock and poultry breeding. TC mainly inhibits the activity of Gram-negative bacteria by binding to the A site of bacterial ribosomal subunits. When they are taken up by bacterial cells, they inhibit protein synthesis by preventing the coupling of aminoacyl to the A-position tRNA. It eventually leads to the death of Gram-negative bacteria including methanogens [11, 12]. Therefore, if there is a certain concentration of residual antibiotics in the feces, it may lead to the collapse of the anaerobic digestion system. When the concentration of TC in cow dung was 10 mg/L, the CH_4_ production was reduced by 7.8% compared with the reactor without TC [13]. It can be speculated that TC pairs may adversely affect methane production in anaerobic digestion, but the effect of anaerobic digestion using chicken manure as a single substrate is not clear.

### 3.2. Calculation of Methane Production

The biogas produced by each treatment group is analyzed according to the gas production every 1–3 days, and the methane production is calculated as follows:

(1) $$\begin{array}{c} V_{CH_{4}}=V_{H}\cdot \Delta C_{CH_{4}}+V_{S}\cdot C_{CH_{4}}, \end{array}$$

where V_CH_4__ is the volume of methane (mL), *V*_*H*_ is the headspace volume (mL), *V*_*S*_ is the amount of gas measured by a syringe (mL), ΔC_CH_4__ is the change in methane concentration (%), and C_CH_4__ is the methane content in the gas (%) [14, 15]. The cumulative methane production is the cumulative methane production of each treatment group − the cumulative methane production of inoculated sludge.

#### 3.2.1. Fitting Model

In order to further explore the influence mechanism of chicken manure mesophilic anaerobic digestion, this study adopts the modified Gompertz model to analyze the kinetic parameters of the cumulative methane curve [16, 17].

(2) $$\begin{array}{c} Y_{\left(t\right)}=M_{m}\cdot \;\exp\left\{-\exp\left[\frac{R_{m}\cdot e}{M_{m}}\cdot \left(\lambda -t\right)+1\right]\right\}. \end{array}$$

#### 3.2.2. Cumulative Hydrolysis, Acidification, Acetation, and Methanation Calculations

In the process of anaerobic digestion, organic matter is sequentially hydrolyzed, acidified, acetic acidized, and finally converted into methane [18]. In a fully mixed system, these four stages cannot achieve process separation. The total amount of accumulated hydrolysis, acidification, acetic acidation, and methanation in the anaerobic digestion process can be calculated by formulas (4)–(6), respectively.

(3) $$\begin{array}{c} C_{\text{hydr}}=\left(\frac{{\text{V}}_{\text{CH}4}}{350}+C_{\text{SCOD}}\cdot \text{V}\right)\cdot {\text{COD}}_{\text{add}}^{-1}, \end{array}$$

(4) $$\begin{array}{c} {\text{C}}_{\text{Acid}}=\left(\frac{{\text{V}}_{\text{CH}4}}{350}+{\text{C}}_{{\text{VFA}}_{S}}\cdot \text{V}\right)\cdot {\text{COD}}_{\text{add}}^{-1}, \end{array}$$

(5) $$\begin{array}{c} C_{\text{Acet}}=\left(\frac{{\text{V}}_{\text{CH}4}}{350}+C_{\text{acctate}}\cdot \text{V}\right)\cdot {\text{COD}}_{\text{add}}^{-1}, \end{array}$$

(6) $$\begin{array}{c} C_{\text{meth}}=\frac{{\text{V}}_{\text{CH}4}}{350}\cdot {\text{COD}}_{\text{add}}^{-1}. \end{array}$$

The cumulative amount of hydrolysis, acidification, acetic acidation, and methanation during anaerobic digestion is represented by the cumulative curve of each process based on SCOD [19]. In the formula, V_CH4_ is the cumulative methane production volume, mL; 350 is the conversion factor for converting the volume of V_CH4_ to SCOD mass; *C*_SCOD_ is the concentration of SCOD, *g·L*^−1^.

### 3.3. Energy Generation

Energy production (Eo) is calculated from methane production according to the following formula:

(7) $$\begin{array}{c} E_{0}=\frac{P_{\text{CH}4}\cdot V\cdot \varepsilon \cdot \eta_{m}}{Q\cdot \text{COD}}. \end{array}$$

where *P*_CH4_ is the output of methane, *L*(*L·d*)^−1^. COD is the concentration of organic matter in the matrix.

(1) In this study, the energy consumption (*E*_*p*_) of the peristaltic pump during the conveying process of substrate discharge and digestive juice discharge was calculated according to the effect of TC on anaerobic digestion of chicken manure under the continuous test conditions of the following formula:
  (8) $$\begin{array}{c} E_{p}=\frac{Q_{p}\cdot \gamma \cdot h}{1000q\eta }\frac{1}{Q\cdot \text{COD}}, \end{array}$$
   where *Q*_*p*_ is the discharge flow rate of the digestive juice; *γ* is 9800 N/m^3^; *h* is the hydraulic pressure head; *q* is the flow rate of matrix discharge, and the flow rate of digestive juice discharge is equal to the flow rate of matrix discharge; and *η* is the efficiency of the pump, which is 60%.
(2) The energy consumption (En) of the agitator for mixing the substrate tank and the fermenter material is calculated according to the formula:
  (9) $$\begin{array}{c} E_{b}=\frac{N_{p}\rho }{10^{6}q\iota }{\left(\frac{n}{60}\right)}^{3}D^{5}\frac{1}{Q\cdot \text{COD}}. \end{array}$$
(3) The energy consumption (En) for raising the water temperature to the temperature in the water bath is calculated according to the formula:
  (10) $$\begin{array}{c} E_{h}=\frac{pQk\cdot \left(T_{d}-T_{a}\right)}{Q\cdot \text{COD}}, \end{array}$$
   where *p* represents the density of the influent water, 1000 kg*∗*m^−3^; *k* represents the specific heat of the influent water, which is 4.18 kJ (kg*∗*C)^−1^; *T*_*d*_ represents the reactor operating temperature, which is 35°C; and *T*_*a*_ represents the ambient temperature, which is 20°C.
(4) In En, about 80% of the heat can be recycled, so the heat recovery rate (*E*) is 80% of that of En. The heat loss (*E*) due to incomplete mass transfer in the reactor is about 5% of En.

### 3.4. Energy Balance

To evaluate the energy balance, the net energy potential (NEP), the energy ratio (*R*_*e*_), and the energy conversion efficiency (*n*) of organic matter are calculated according to formulas (11)–(13), respectively:

(11) $$\begin{array}{c} \text{NEP}=E_{0}-\left(E_{p}+E_{b}+E_{h}-E_{r}+E_{1}\right), \end{array}$$

(12) $$\begin{array}{c} R_{e}=\frac{E_{0}}{E_{p}+E_{b}+E_{h}-E_{r}+E_{1}}, \end{array}$$

(13) $$\begin{array}{c} \eta_{s}=\frac{\text{NEP}}{Q\cdot \text{COD}\cdot R_{s}}, \end{array}$$

where *R*_*s*_ is the COD removal rate.

### 3.5. 3D-EEM Fluorescence Spectrum Analysis and Fluorescence Area Integration Analysis

3D-EEM spectral data analysis was performed using FRI technology. The 3D-EEM spectral data were analyzed by FRI technique, and the volume of EEM region “*i*” was Φ_*i*_, and the normalized region volume (Φ_*i*,*n*_, Φ_*T*,*n*_) for different excitation/emission wavelengths was calculated with the following formula:

(14) $$\begin{array}{c} \Phi_{i,n}={\text{MF}}_{i}\Phi_{i}={\text{MF}}_{i}\sum_{ex}\sum_{em}Ι\left(\lambda_{ex}\lambda_{em}\right)\Delta \lambda_{ex}\Delta \lambda_{em},\\ \Phi_{Τ,n}=\sum \Phi_{i,n}, \end{array}$$

where Δ*λ*_*ex*_ is the excitation wavelength interval (5 nm) and Δ*λ*_*em*_ is the emission wavelength interval (5 nm).

The percent fluorescence response (*P*_*i*,*n*_, %) is calculated by:

(15) $$\begin{array}{c} P_{i,n}=\frac{\Phi_{i,n}}{\Phi_{i,n}}\times 100\%. \end{array}$$

## 4. Anaerobic Digestion of Chicken Manure with Tetracycline Antibiotics

### 4.1. Experimental Samples and Characteristics

The inoculated sludge was taken from the continuous and stable operation of the medium-temperature anaerobic digester of Xi'an Peimin Co., Ltd. The characteristics of the materials are shown in Table 1.

As shown in Table 1, fresh chicken manure was taken from the Huifeng Poultry Industry Black-Bone Chicken Breeding Base in Yangling Demonstration Zone, Shaanxi Province, and the chicken feathers and stones were removed and stored in a −18°C refrigerator for later use. The antibiotic TC (purity 98.0%, CAS NO.64-75-5) used in this study was purchased from Beijing Bailingwei Technology Co., Ltd.

### 4.2. Changes in Methane Production from Anaerobic Digestion of Chicken Manure under Different TC Concentrations

The biochemical methane potential (BMP) experiment used a 100-mL serum bottle with an effective volume of 60 mL. Seven groups of treatments were set up in the experiment: *R*0–*R*6, where *R*0 was the control group. The batch experimental design is shown in Table 2.

As shown in Table 2, in this study, only inoculated sludge was added to the CK treatment group in the empty group to eliminate the effect of gas production from inoculated sludge. Before adding chicken manure, it is diluted to about 4% TS with an appropriate amount of distilled water, mixed with the inoculated sludge at a ratio of 1 : 3, and added with different concentrations of TC. It regularly collects fermentation broth and conducts targeted determination of its physical properties, and it regularly measures fermentation broth, gas production, and gas composition.  Figure 1 shows the batch test equipment and how to measure the amount of gas produced.

As shown in Figure 1, in order to ensure anaerobic conditions, the serum bottle was flushed with nitrogen gas for 3 min before the experiment. The serum bottle was placed in a constant temperature water bath shaking box at 35 ± 1°C, and the gas production and gas composition were measured regularly. All treatments were set up in 3 replicates.

### 4.3. Effects of TC on Dissolution, Hydrolysis, Acidification, and Methanation

Anaerobic digestion usually goes through four processes: dissolution, hydrolysis, acidification, and methanation. In previous studies, the effects on the reaction rate of the dissolution process were usually obtained by batch experiments with actual substrates as substrates, and the reaction rates of hydrolysis, acidification, and methanation were usually batch experiments with model substrates. Therefore, batch experiments using chicken manure or synthetic wastewater will be conducted to evaluate the effect of TC on dissolution, hydrolysis, acidification, and methanation processes. In this experiment, twenty-one 100-mL serum bottles were divided into three experimental groups (Experiment I, Experiment II, and Experiment III). Each experimental group was further divided into 7 treatment groups. It used Experiment I, Experiment II, and Experiment III to evaluate the effect of TC on hydrolysis, acidification, and methanation, respectively. All experiments lasted 3 days.

For the dissolution process, it was sampled within the optimal digestion time (3 days). It measures the concentration of soluble protein and polysaccharide in the fermentation broth and analyzes the components of its EPS in combination with three-dimensional fluorescence.

### 4.4. The Effect of Anaerobic Fermentation of Chicken Manure with TC Concentration on Methane Content

The daily methane production of chicken manure anaerobic fermentation with different TC concentrations under sequencing batch test conditions is shown in Figure 2.

It can be seen from Figure 2 that the daily methane production with different TC concentrations first increased and then decreased gradually. It is mainly due to the hydrolysis and acidification of easily degradable organic matter such as carbohydrates and proteins in the early stage of fermentation, and the produced VFAs are utilized by methanogens. Therefore, the gas production at each stage gradually increased, followed by the consumption of easily degradable VFAs. The daily methane production at each stage dropped rapidly. It shows that the gradual domestication of the sludge is realized by the method of adding TC in stages by the sequencing batch test, so that the anaerobic microorganisms can enhance the tolerance to toxicity.

## 5. Results of Anaerobic Digestion of Chicken Manure

### 5.1. Effect of TC on Methane Production from Anaerobic Digestion

The methane production of anaerobic digestion when adding different concentrations of TC in this study is shown in Figure. It can be seen that the methane production varies significantly with time from 0 to 9 days, but the increase is smaller until the end of the anaerobic digestion. The daily methane production and cumulative methane production of *R*0–*R*6 are shown in Figure 3.

As can be seen in Figure 3, only a small amount of gas was produced in each treatment group on the first day of anaerobic digestion. It may be because the microorganisms have not yet adapted to the new anaerobic digestion environment. But on the third day after the start of the experiment, with the rapid decomposition of organic matter, all experimental groups reached the peak of methane production without a significant lag period. The methane yields of the *R*0–*R*6 groups were 44.68, 49.68, 46.84, 45.81, 46.97, 44.91, and 42.09 mL, respectively. It may be due to the rapid decomposition of easily degradable organic matter at this time, resulting in the first peak of gas production. A second small peak of methane production in each group (except *R*6) could be observed on day 6. However, there was a lag period in the methane production of the *R*6 group, and the second small peak appeared on the 7th day. It may be due to the hydrolysis of nondegradable organics in the substrate at this time, resulting in a slight increase in methane production. From the 9th day to the end of anaerobic digestion, the methane production in each group decreased significantly until the gas production stopped. This is because the organic matter in the substrate is consumed during the digestion process, resulting in insufficient nutrients for the microorganisms to use, so the methane production continues to decline. At the end of the test, the cumulative methane production of the *R*1–*R*6 groups was 208.88, 210.71, 203.63, 207.54, 207.55, and 190.87 mL, respectively, and the control group was 203.44 mL. The methane production of *R*2 increased by about 3.57% compared with the control, while the methane production of *R*6 decreased by 12.57 mL, and the inhibition rate was 6.18% (*P* < 0.05). The correlation coefficient (*R*2) is shown in Table 3.

As shown in Table 3, the maximum cumulative methane production Mm is (202.08 ± 1.70 mL) > *R*1 (200.29 ± 1.78 mL) > *R*5 (200.16 ± 1.57 mL) > *R*4 (199.68 ± 1.64 mL) > *R*3 (196.64 ± 1.52 mL) > *R*0 (195.51 ± 1.74 mL) > *R*6 (183.64 ± 1.38 mL). The maximum methane production rate Rm is in the order of *R*4 > *R*1 > *R*0 > *R*2 > *R*3 > *R*5 > *R*6. It shows that a TC concentration of 300 mg/L has an inhibitory effect on methanogenesis and methanogenesis rate.

### 5.2. Effects of TC on PH and VFA in Anaerobic Digestion

The initial pH value of all treatment groups was between 7.56 and 7.78, which was the suitable pH range for anaerobic digestion. From day 3 to day 7 of anaerobic digestion, pH was gradually increased in all treatment groups. The pH values of *R*0–*R*6 increased from 7.56, 7.5, 7.5, 7.44, 7.43, 7.37, 7.41, 7.39, and 7.35 to 7.78, 7.79, 7.74, 7.76, 7.75, 7.76, 7.74, 7.7, and 7.72, respectively. Possibly because it is in the first stage of anaerobic digestion at this time, the organic substrate is anaerobic biodegraded to form protein, urea, etc., resulting in an increase in pH value. Subsequently, under the action of hydrogen-producing acetogens, it converts the early intermediates in the digestive system into VFAs, H_2_, and CO_2_. The system began to produce and accumulate acid, resulting in a gradual decrease in pH in each treatment group. Changes in *R*0–*R*6 pH and VFA are shown in Figure 4.

As shown in Figure 4, VFAs are intermediates in the degradation process of anaerobic digestion. The VFA concentrations of each treatment group reached the maximum on day 2, which were 840.98, 967.80, 872.57, 636.71, 683.62, 652.22, and 560.61 mg/*g* VS, respectively. It may be because the easily degradable 630 organics are rapidly dissolved and hydrolyzed. As the organic matter was continuously depleted, VFA production continued to decline in all treatment groups until the end of anaerobic digestion. The VFA concentrations of *R*0–*R*6 were 35.58, 38.23, 36.85, 35.96, 36.01, 40.12, and 37.44 mg/*g* VS, respectively. There was no significant difference in the content of all treatment groups, and no acid accumulation occurred. This change phenomenon is similar to the change in daily methane production. The massive production of VFA enables methanogens to rapidly convert it into methane, resulting in a rapid peak of methane production 3 days before anaerobic digestion. As the production of VFA decreases, the methanogens have no available substrate, resulting in a continuous decline in methane production. The changes in *R*0–*R*6 pH and VFA are shown in Figure 5.

As can be seen in Figure 5, the increase in VFA production in the *R*0–*R*6 group on day 2 of anaerobic digestion was mainly due to the increase in acetate and propionate. It is inferred from this that the type of anaerobic fermentation of chicken manure is acetic acid fermentation, and the concentration of acetic acid accounts for 37.68%∼49.30% of the total concentration of VFAs. On the fourth day of the reaction, acetic acid was rapidly consumed in each treatment group, while the concentration of propionic acid increased slightly. It may be because propionic acid cannot be directly used by microorganisms to produce methane, so that propionic acid needs to be converted into acetic acid before it can be used by microorganisms. As the reaction progressed, the organic acid concentration of each treatment group gradually decreased. Only trace amounts of acetic acid were present in the system until the end of the reaction. The acetic acid degradation rates of R0–R6 were 90.58%, 89.63%, 89.67%, 85.01%, 86.22%, 86.76%, and 86.45%, respectively.

### 5.3. Effect of TC on the Dissolution Process of Anaerobic Digestion

Anaerobic digestion usually includes the four processes of dissolution, hydrolysis, acidification, and methanation. In order to understand the effect of TC on each process, this article studies the effect of TC on each process. The effects of TC on soluble polysaccharides and proteins are shown in Figure 6.

As shown in Figure 6, all TC-added treatment groups had no obvious effect on the content of soluble protein, but the content of polysaccharide had obvious changes. Compared with the control group, adding 25 mg/L of TC increased the polysaccharide content by 29.03 mg COD/L, and the concentration of TC at 300 mg/L had the highest inhibition rate, which was 27.03% lower than that of the control group. This suggests that low concentrations of TC can promote the solubilization of digestive substrates, which is consistent with other antibiotics such as CLA. Previous studies have shown that the addition of antibiotics can promote the rupture of anaerobic digestion cells, thereby accelerating the hydrolysis of anaerobic sludge. The effect of TC on hydrolysis is shown in Figure 7.

As shown in Figure 7, similar to the dissolution stage, the change in TC on the degradation efficiency of BSA was negligible, but the effect on the degradation efficiency of glucan was quite significant. When TC was added at 25 mg/L, the degradation efficiency of glucan was 65.12%. When the concentration of TC was 300 mg/L, the degradation efficiency of glucan reached the lowest level, which was only 2.95%. It shows that high concentration level of TC has inhibitory effect on the degradation of glucan, and the inhibitory effect is more obvious when the concentration is higher. The effect of TC on the acidification process was investigated by the determination of VFAs in the samples as shown in Figure 8.

As shown in Figure 8, it can be seen that when the TC concentration is 25 mg/L, the lowest VFAs production is 32.77 mg COD/L, which is about 26.54% lower than that of the control group. However, when the concentration was 300 mg/L, there was no significant change compared with the control group. The VFAs produced during anaerobic digestion are consumed during methanation to produce CH_4_. Therefore, the inhibition of the methanation process may also lead to the accumulation of VFAs. Conversely, the decrease in VFAs caused by the addition of TC may be due to its promotion of methanogenesis. For validation, we assessed the effect of TC on methanogenesis. The results showed that the maximum methane production was 15.23 mL when 25 mg/L TC was added in this study, which is an increase of 1.84 mL compared with 13.39 mL in the control group. This result confirmed the above possibility that TC led to the reduction of VFAs production because it promoted the production of CH_4_, thereby depleting the content of VFAs in the digestive system.

### 5.4. Effect of TC on EPS

EPS is a natural biopolymer with diverse structures and components, and polysaccharides and proteins are its main components. EPS is an organic substance secreted by microorganisms that attaches to the sludge cells as an anticoagulant to protect the cells from toxic substances. It can therefore be hypothesized that the increase in carbohydrate content may be due to TC-promoting EPS secretion. To test this hypothesis, the changes in LB-EPS and TB-EPS contents were investigated as shown in Figure 9.

As shown in Figure 9, it can be seen that 25 mg/L of TC significantly increased the content of LB-EPS and also had a certain promotion effect on the secretion of TB-EPS. Consistent with previous studies, the addition of antibiotics stimulated EPS secretion.

The compositional changes in LB-EPS and TB-EPS are shown in Figure 10.

As shown in Figure 10, in LB-EPS, the humic acid-like and fulvic-like acids (components of humic substances) in the TC-added treatment group were higher than those in the control group. It shows that at low concentrations (10, 25 mg/L), TC mainly promotes the degradation of LEPS by promoting the dissolution of intracellular substances in the sludge. With the increase of TC concentration (50–300 mg/L), TC mainly promotes the breakdown of the sludge cell membrane by promoting the rupture of the sludge cell membrane, thereby promoting the degradation of LEPS. There was no significant change in the content of various substances compared with the control group. It shows that the addition of TC did not have any effect on the proportion of bound EPS, as well as the organic matter and organic matter components. This may be because TB-EPS acts as the inner core host of the EPS dense network structure. It adheres to the surface of microbial cells and is difficult to be degraded.

### 5.5. Effects of TC on HIX and FI in EPS

The fluorescence index (FI) was used to determine the source of humic-like organic matter in the sample. The HIX and FI of the three types of EPS in the *R*0–*R*6 treatment group are shown in Table 4.

It can be seen from Table 4 that in the S-EPS, the HIX values of the *R*1–*R*5 groups basically did not change. The HIX value of the *R*6 group was 0.60, slightly higher than the control group's 0.48. In LB-EPS, the HIX value of the *R*2 group (0.29) was 0.14 lower than that of the control group *R*0 (0.43). However, the HIX of all treatment groups in TB-EPS was basically the same. It shows that when the TC concentration is 25 mg/L, the humification degree of EPS is generally low, and the organic matter becomes unstable and more easily utilized by microorganisms. When a high concentration of TC (300 mg/L) was added, the degree of humification of EPS was high, and it was not easy to be utilized by microorganisms. FI ≤ 1.4 indicates that the humic organic matter in the sample comes from the matrix itself, and FI ≥ 1.9 indicates that the humic organic matter in the sample is a microbial derivative. The FI values of the three EPSs in all the treatment groups were lower than 1.4, indicating that all humic substances were derived from the substrate itself, and not from microbial-derived substances.

## 6. Conclusion

In this experiment, the effect of tetracycline on the anaerobic digestion of chicken manure was studied to understand the inhibition limit of tetracycline on the anaerobic digestion of chicken manure. Combined with the analysis of EPS and 3D-EEM, the mechanism of tetracycline inhibiting anaerobic fermentation of chicken manure was discussed. The results showed that anaerobic digestion microorganisms were inhibited when a high concentration of TC (300 mg/L) was added. This study can provide evidence for the effect of anaerobic digestion of TC-containing chicken manure. This is critical for handling antibiotic-laden chicken manure waste. The single-factor analysis method was adopted in this experiment, and only the effects of different concentrations of TC and biochar on the anaerobic fermentation of chicken manure were investigated, but the important factors such as pH, temperature, mixing ratio, CN, substrate concentration, and other important factors on the anaerobic fermentation of chicken manure were not further studied. The optimal conditions for anaerobic fermentation of chicken manure for methane production were obtained.

## Figures and Tables

**Figure 1:** Batch test device and gas generation measurement.

**Figure 2:** The daily output of methane in anaerobic fermentation of chicken manure with TC concentration.

**Figure 3:** Daily methane production and cumulative methane production of *R*0–*R*6. (a) Daily methane production. (b) Cumulative methane production.

**Figure 4:** Changes in pH and VFA in *R*0–*R*6.

**Figure 5:** Changes in pH and VFA in *R*0–*R*6. (a) *R*0, (b) *R*1, (c) *R*2, (d) *R*3, (e) *R*4, (f) *R*5, and (g) *R*6.

**Figure 6:** The effect of TC on soluble polysaccharides and proteins. (a) The effect of TC on soluble polysaccharides. (b) The effect of TC on proteins.

**Figure 7:** Lysate (dextran) and lysate degradation (BSA). (a) Degradation of lysate (dextran). (b) Degradation of lysate (BSA).

**Figure 8:** Changes in acidified product (VFA) and acidified product methane production. (a) Change in acidification product (VFA). (b) Change in methane production in acidification product.

**Figure 9:** Changes in LB-EPS and TB-EPS contents.

**Figure 10:** Compositional changes in LB-EPS and TB-EPS.

**Table 1:** Physicochemical properties of inoculated sludge and fresh chicken manure.

Analytical parameters	Unit	Chicken manure	Inoculum sludge
Total solids (TS)	%	32.9	3.16
Volatile solids (VS)	%	25.4	1.42
Total chemical oxygen demand (TCOD)	mg/L	51066.67	21366.67
Total protein	mg/L	41136.36	4636.36
Polysaccharide	mg/L	10642.86	7857.14
pH	—	7.05	8.09
TC	mg/kg	0	0

**Table 2:** Batch experimental design.

NO.	Manure (mg)	Inoculum (mg)	TC (mg)
*R*0	15	45	0
*R*1			0.15
*R*2			0.375
*R*3			0.75
*R*4			1.125
*R*5			2.25
*R*6			4.5
CK	0	45	0

**Table 3:** The modified Gompertz formula to simulate the cumulative methane production curve.

Key parameters	Mm (mL)	Rm (mL)	*λ* (d)	*R*2
*R*0	195.51 ± 1.74	37.36 ± 2.19	0.42 ± 0.16	0.99
*R*1	200.29 ± 1.78	37.83 ± 2.19	0.39 ± 0.16	0.99
*R*2	202.08 ± 1.70	36.51 ± 1.94	0.33 ± 0.16	0.99
*R*3	196.64 ± 1.52	36.29 ± 1.80	0.36 ± 0.14	0.99
*R*4	199.68 ± 1.64	37.87 ± 2.03	0.48 ± 0.15	0.99
*R*5	200.16 ± 1.57	34.82 ± 1.68	0.31 ± 0.15	0.99
*R*6	183.64 ± 1.38	31.12 ± 1.40	0.42 ± 0.14	0.99

**Table 4:** HIX and FI of three types of EPS in *R*0–*R*6 treatment group.

	*R*0	*R*1	*R*2	*R*3	*R*4	*R*5	*R*6
S-EPS							
HIX	0.48	0.52	0.47	0.50	0.53	0.51	0.60
FI	0.81	0.82	0.82	0.82	0.82	0.82	0.81

LB-EPS							
HIX	0.43	0.38	0.29	0.35	0.29	0.34	0.45
FI	0.82	0.82	0.82	0.82	0.82	0.81	0.82

TB-EPS							
HIX	0.29	0.29	0.29	0.30	0.35	0.30	0.31
FI	0.81	0.82	0.82	0.82	0.82	0.82	0.82

## Data Availability

No data were used to support this study.
